# Analysis of the Influence of Midwife Led Antenatal Clinic on the Delivery Outcomes of Primipara under the Evaluation of Medical Data

**DOI:** 10.1155/2022/7454258

**Published:** 2022-10-11

**Authors:** Wei Fan, Ling Wang, Lili Zhang, Xiaoling Liu, Zhaoyan Meng

**Affiliations:** Department of Obstetrics, Gansu Provincial Maternity and Child-care Hospital, Lanzhou, 730050 Gansu, China

## Abstract

**Objective:**

In order to improve the comprehensive effect of primipara delivery outcomes, the midwife led prenatal clinic of data mining is analyzed to alleviate the negative emotions of patients and improve the delivery results of patients.

**Methods:**

A total of 86 patients who were filed in the obstetrics department of our hospital from October 2021 to May 2022 and planned to deliver in our hospital were selected as the research objects. They were divided into the reference group (*n* = 43) and the observation group (*n* = 43) according to the random number table method. Among them, the reference group received routine antenatal clinics, and the observation group received midwives' participation in antenatal clinics for intervention. The total duration of labor, the scores of various psychological states including antenatal anxiety (SAS) and antenatal depression (SDS), as well as the pregnancy outcome and delivery compliance rate of the two groups were compared.

**Results:**

The psychological state evaluation of delivery in the observation group, whether SAS score or SDS score, was significantly lower than that in the reference group, and the difference was statistically significant. The whole labor process time of patients in the observation group was significantly shorter than that in the reference group, and the difference was statistically significant. The delivery compliance of patients in the observation group during the whole perinatal period was also higher than that of the reference group, and the difference was statistically significant. All *P* values were<0.05.

**Conclusion:**

The antenatal clinic led by midwives can promote primiparas to increase the success rate of natural delivery, improve the treatment compliance of the whole perinatal period, reduce the psychological pressure of primiparas, effectively shorten the total time of production, and have a significant impact on the outcome of delivery. It should be widely used.

## 1. Introduction

In order to improve the informatization construction level of Obstetrics and Gynecology and the efficiency of using massive case diagnosis and treatment data, through the in-depth analysis of the general data of patients, the big data processing technology can analyze the diagnosis and treatment decisions of Obstetrics and Gynecology and the health indicators of Obstetrics and gynecology patients, and the data mining technology can use genetic algorithm to preliminarily judge the health status of primiparas and newborns from the medical database, The diagnosis results will be transmitted to the cloud database in real time, so that midwives can understand the health of pregnant women and fetus in real time. Data mining algorithm in maternal and fetal signs information analysis, if abnormal parameter indicators occur, we can give help in time and buy valuable time for newborns. If you want to give birth smoothly, pregnant women need to master the necessary scientific knowledge during pregnancy and make full preparations before delivery. The antenatal clinic led by midwives should actively publicize the benefits of natural childbirth, establish confidence in natural childbirth and promote natural childbirth. Xiyao [1] used midwife psychological nursing intervention to significantly reduce the probability of primiparas choosing cesarean section in the whole perinatal care of primiparas. Psychological nursing intervention can improve the bad mood of primiparas, shorten the whole labor process, and promote the newborn to be healthier [1]. Suqing et al. [2] analyzed that the role standardized progressive nursing model can alleviate primiparas' fear of delivery, improve their sense of delivery self-efficacy, and improve the outcome of delivery. Ruilan and Ruiju [3] can shorten the time of the first and second stages of labor, improve the anxiety and depression of primiparas, and promote the natural delivery rate of primiparas by implementing midwife psychological intervention on primiparas. Pei [4] pointed out that the midwife led pelvic swing intervention in the delivery process of primiparas can effectively shorten the time of each stage of labor and the total stage of labor, alleviate the degree of pain in the process of labor, improve the negative psychology of primiparas, and the application effect is obvious. Ying [5] made primiparas understand the whole process of production through the intervention of animated video of delivery education. When they rely on their mastered delivery knowledge in the process of production, they can adjust their negative emotions, reduce the pain of the whole delivery, and improve the delivery outcome of primiparas.

Suqin [6] and others discussed that clinical medical staff should pay attention to the cultivation and intervention of the positive psychological level of primiparas, which can improve the health literacy level of primiparas throughout the perinatal period, alleviate the fear of delivery, and reduce the incidence of cesarean section. Jun [7] analyzed the application of data mining technology in medical big data in terms of association rule mining, classification mining, cluster analysis, etc. through data mining technology, providing a good environmental support for data mining technology. Gang [8] analyzed that with the development of hospital informatization, medical big data has shown explosive growth. Using data mining technology, medical business information is classified and processed, and the digitalization of information management improves the overall service quality of the hospital, which can fully mine the hidden parameters in information management, so as to improve the management level of the hospital [8]. Yan [9] pointed out that the prenatal clinic led by midwives can effectively improve the negative emotions of primiparas during pregnancy and delivery, improve the natural delivery rate, and reduce the influencing factors of cesarean section.

By comparing two different groups of antenatal clinics, the antenatal clinic led by midwives can adjust the psychological state of patients, reduce the degree of depression and anxiety of patients, and relieve the negative emotions of patients. Under the data depth mining technology, through technical analysis and provide precautions corresponding to the gestational age, and carry out health education, popularize childbirth knowledge to patients, let patients know and understand, so as to improve the outcome of childbirth.

## 2. Data and Grouping

### 2.1. General Information of Patients

86 pregnant women who were filed in the obstetrics department of our hospital from October 2021 to May 2022 and planned to deliver in our hospital were selected as the research objects. In this study, random number table method was used to randomly divide into reference group and observation group. 43 patients in the reference group received routine antenatal clinics and 43 patients in the observation group received midwife led antenatal clinics on the basis of the reference group. The age of the reference group was 20 to 34 years old, the average age was (25.7 ± 1.8) years old, the gestational weeks were 28 to 40 weeks, the average gestational weeks were (34.3 ± 2.8) weeks, and the average weight was (69.2 ± 3.8) kg. The age of the observation group was 21 to 34 years old, the average age was (26.5 ± 2.1) years old, the gestational weeks were 29 to 41 weeks, the average gestational weeks were (35.5 ± 1.7) weeks, and the average weight was (70.9 ± 4.3) kg.

### 2.2. Inclusion and Exclusion Criteria

#### 2.2.1. Inclusion Criteria

1. Primipara, intrauterine singleton, term pregnancy
2. Pelvic measurement, fetal position examination and B-ultrasound monitoring are all in the normal range
3. Have normal communication skills
4. Know and agree with this study

#### 2.2.2. Exclusion Criteria

1. Severe pregnancy complications
2. Maternal patients older than 35 years old
3. Patients with contraindications
4. Abnormal conditions occur in the process of prenatal examination during pregnancy

### 2.3. Observation Indicators

1. The SAS scores of the two groups were observed and recorded
2. Observe and record the SDS scores of the two groups of patients
3. Observe and record the results of labor process time
4. Observe and record the delivery outcome of the two groups of patients
5. Observe and record the delivery compliance of the two groups of patients

## 3. Method

### 3.1. Routine Antenatal Clinic (Reference Group)

The reference group asked the pregnant woman's medical history in detail during the antenatal examination; give routine prenatal education; regularly measure blood pressure and weight; regular monitoring of routine hematuria and blood biochemistry; conduct standard fetal heart rate monitoring; and answer the questions of pregnant women.

### 3.2. Antenatal Clinics Attended by Midwives (Observation Group)

On the basis of routine antenatal outpatient care in the observation group, data mining technology and data analysis software are used to collect and analyze the information of past cases, so as to draw a reasonable and feasible process map of pregnancy care and provide appropriate antenatal outpatient services for primiparas. According to the nursing progress chart during pregnancy, midwives (1) record the history and requirements of pregnant women from 26 to 32 weeks of pregnancy, and establish a good doctor-patient relationship with pregnant women and their families; educate pregnant women about the importance of weight control, and formulate a personalized healthy diet plan according to the nutritional status of pregnant women; (2) from the 33rd to 35th weeks of pregnancy, explain to pregnant women when to choose hospitalization, and inform pregnant women and their families to prepare items before delivery; show pregnant women the real picture of the delivery room and relevant videos to help them understand the environment of the delivery room; (3) at the 36th week of pregnancy, according to the actual situation of pregnant women, inform pregnant women of the labor process, the selection factors of delivery methods, the process of natural delivery and cesarean section, as well as the advantages and disadvantages of various delivery methods, and guide pregnant women to exercise appropriately; guide the pregnant woman's husband's paternity work; and (4) from the 37th week of pregnancy to the time of delivery, popularize knowledge about postpartum health care and neonatal nursing skills to pregnant women and their families. During this period, big data mining technology is used to collect and count the problems that affect pregnant women's emotions. Through the analysis results, it was found that direct and effective psychological counseling and doubt elimination are implemented for pregnant women to reduce their psychological pressure.

### 3.3. Statistical Methods

The research conducted information grouping analysis according to statistical software, and compared the data association basis and corresponding relationship of different information of the two groups of research objects. The specific statistical methods used are measurement data: statistics are given by means of mean ± standard deviation; counting data: percentage counting method; and the measurement data between the two groups were compared by *t*-check method, and the counting data were compared by chi square test. The correlation analysis test method of the related variables of the two groups of objects was used. *P* < 0.05, the difference was statistically significant.

## 4. Simulation Verification

### 4.1. SAS Score and SDS Score Analysis of Primiparas in the Two Groups

Most primiparas will appear varying degrees of anxiety, depression, panic, and other emotions in the perinatal period. Due to the lack of delivery experience, insufficient knowledge of delivery, and the perinatal mental state, they play a decisive role in the process of delivery. In the process of delivery, they always maintain a state of tension and panic, which is easy to lead to uterine contraction. The antenatal clinic dominated by midwives needs to inform primiparas of the precautions to keep primiparas in a positive state. Now the scoring results of the two groups of primiparas, and the following Table 1 is obtained.

Table 1 shows the psychological state evaluation results of the two groups of primiparas. After investigating and analyzing the SAS and SDS scores of the patients, it can be seen that the anxiety and depression of the patients in the reference group are higher than those in the observation group, which indirectly shows that the prenatal clinic led by midwives can improve the psychological state and bad mood of the patients.

In order to better analyze and compare the psychological status of the two groups of primiparas, the following Figure 1 is obtained by visualizing the data in Table 2.

As shown in Figure 1, the visualization effect of the comparative data of the two groups of primiparas is shown. The psychological state of the patients in the observation group is better than that of the patients in the reference group. It can be concluded that the prenatal clinic led by midwives can help patients adjust their state.

### 4.2. Comparison of the First and Second Stages of Labor between the Two Groups of Primiparas

The antenatal clinic led by midwives can give patients and their families knowledge about pregnancy and childbirth, actively answer their questions and concerns, adjust and change some wrong behavior perceptions of primiparas and their families, and carry out health education for primiparas to tell the advantages and disadvantages of different delivery methods, so as to meet the knowledge needs of primiparas, Let primiparas better understand the benefits of natural childbirth for themselves and newborns, and on this basis, use data mining technology to evaluate the risk of natural childbirth of primiparas, and help them build confidence in natural childbirth. Now compare the labor process time of the two groups of primiparas, and make a chart according to the recorded results, and get the following Table 2.

Table 2 shows the time comparison results of the first stage of labor and the second stage of labor of the two groups of primiparas. From the data results, the midwife led prenatal clinic can help them understand the whole production process and effectively shorten the length of production.

In order to better compare the labor process time of the two groups of primiparas, the following Figure 2 is obtained by visualizing the data in Table 3.

As shown in Figure 2, the visualization effect of the comparison of labor process time between the two groups of primiparas is shown. The total labor process of primiparas in the observation group was significantly lower than that in the control group, which indirectly showed that the prenatal clinic dominated by midwives could shorten the labor process.

### 4.3. Comparison of Delivery Outcomes between the Two Groups of Primiparas

Labor is accompanied by labor pains, which will bring great pain to primiparas. Primiparas have excess nutrition in the perinatal period, and their weight increases too fast, which will lead to macrosomia. Macrosomia is more likely to have dystocia in the process of delivery, or the method of lateral resection of delivery allows newborns to deliver smoothly. The prenatal clinic led by midwives should strengthen the prenatal health education of patients, eat reasonably, and exercise to control weight, So as to reduce the birth rate of macrosomia. Among them, dystocia, emergency cesarean section and too long labor process will lead to the incidence of cesarean section. Now, the delivery outcomes of the two groups of primiparas are compared, and the chart is made according to the recorded results, and the following Table 3 is obtained.

Table 3 shows the data results of natural delivery, delivery lateral resection, involuntary cesarean section, and voluntary cesarean section of the two groups of primiparas. Prenatal clinics led by midwives have a significant impact on the delivery outcome of primiparas, which can be popularized, improve the delivery rate and the outcome of delivery.

In order to better analyze the delivery outcomes of the two groups of primiparas, the following Figure 3 is obtained by visualizing the data in Table 3:.

As shown in Figure 3, it shows the visual effect of the delivery outcomes of the two groups of primiparas. From the data in the figure, the natural delivery rate of primiparas in the observation group is significantly higher than that of the reference group, which indirectly shows that the prenatal clinic led by midwives can maximize the delivery safety of patients and further improve the natural delivery rate.

### 4.4. Analysis of Survey Results of Production Compliance Rate of Patients

On the basis of big data analysis and in-depth mining, the prenatal clinic led by midwives can not only bring data information support to primiparas but also carry out timely health education in smart medicine. In data mining, regional population prediction and neonatal analysis can be carried out. Big data analysis provides a comprehensive knowledge explanation for primiparas, which can relieve the nervous psychological state of patients, make timely answers to the psychological questions of patients, educate the relevant health care measures of patients with appropriate gestational weeks, and improve the maternal cognition of childbirth through education, so that the maternal can realize the benefits of natural childbirth, and improve the patient's cooperation and compliance with childbirth. On the basis of data mining technology, it is safe to standardize the midwife clinic and make use of mother and baby. Now we compare the delivery compliance rate of the two groups of patients, and make a chart according to the survey results, and get the following Table 4.

Table 4 shows the comparison results of the compliance rates of the two groups of patients in the production process. From the statistical results, the cooperation and compliance of the patients in the observation group in the whole production process are obviously different from that of the reference group. Therefore, it is inferred that the midwife led prenatal clinic of data mining can improve the compliance of patients.

In order to better analyze the delivery compliance rate of the two groups of patients, the following Figure 4 is obtained by visualizing the data in Table 4:

As shown in Figure 4, the visualization effect of the delivery compliance rate of primiparas in the two groups is shown. From the results in the figure, the cooperation compliance rate of primiparas in the observation group is significantly higher than that of the reference group, which indirectly shows that the prenatal clinic led by midwives can provide prenatal guidance to patients and correctly understand delivery pain.

## 5. Discussion

Based on data mining, the health delivery education in antenatal clinic led by midwives can improve the cooperation and compliance of primiparas. Compared with cesarean section, natural delivery is less traumatic to the maternal body, which is conducive to the recovery speed of postpartum body. In addition, it is also beneficial to newborns, which can improve the immune ability of newborns, so as to ensure the health of newborns. Health education before delivery can relieve the panic of unknown and promote the progress of labor to a certain extent. Shaohua and Xiaohua [10] targeted to improve the professional ability of midwifery students and clinical midwives, fully integrate information technology means, and improve the professional ability and level of midwives. Lizhen and Jingdang [11] analyzed that the midwife clinic can improve the outcome of delivery by carrying out the group production education mode, which can help primiparas reduce the stress response better than pain. Improve the psychological state of primiparas and reduce the discomfort of primiparas [11]. The antenatal clinic led by midwives can reduce the occurrence of anxiety and depression of primiparas. Through the antenatal clinic, mothers can realize that their emotions will affect the fetus and help them complete self-emotion regulation. Fengling [12] discussed that the technical level of midwives directly affects the safety of pregnant women and newborns. The prenatal clinic led by midwives is conducive to building a good nurse patient relationship, effectively reducing the amount of postpartum hemorrhage, and shortening the labor process [12]. Huanyuan [13] pointed out that midwifery nursing skills can improve midwives' midwifery skills, further improve primiparas' self-efficacy and delivery control, and improve the impact of delivery outcomes [13]. Lirong et al. [14] discussed the application method and effect of simulated childbirth education combined with individualized psychological counseling in the outpatient nursing of midwives. In the vicinity of childbirth, mothers will more or less have different degrees of anxiety and depression, improve their childbirth cognitive level, and relieve the patient's mood [14]. Fengling pointed out that the level of midwives directly affects the safety of mothers and infants. They can deal with various emergencies that may occur in the process of labor, understand the situation and reactions of mothers, and guide primiparas with midwives' prenatal clinics, which is conducive to improving the effect of labor pains and promoting the progress of labor .

In this study, under the data mining technology, the effect of midwife led antenatal clinic on the delivery outcome of primiparas was deeply discussed. The results showed that the observation group of midwife led antenatal clinic was lower than the reference group in SDS and SAS scores, which could effectively shorten the whole perinatal labor process time, and the delivery compliance was also higher than the reference group. To sum up, the midwife led antenatal clinic based on data mining has high application value.

## 6. Summary

This study focuses on the analysis of data mining technology in the midwife led prenatal clinic to alleviate the negative emotions of patients and improve the outcome of delivery. Through the research of statistical methods, it is found that using data mining technology to extract hidden useful information and rules can more conveniently find the rules between data, predict and evaluate the data that patients conform to the characteristics according to the rules, and there are different analysis methods for different patients, midwives can clearly grasp the nursing process, give practical measures and guidance for the stage of primiparas, directly solve the questions of primiparas, reduce the psychological pressure of primiparas, and effectively improve the outcome of delivery. After the midwife led prenatal outpatient care based on data mining, the SDS and SAS scores of primiparas are lower than those of the conventional prenatal outpatient group. At the same time, the whole labor process is shorter and the delivery compliance is higher, which proves that the midwife led prenatal outpatient care based on data mining is a more ideal method and is worthy of clinical promotion.

## Figures and Tables

**Figure 1:** Visualization of SAS and SDS scores of primiparas in two groups.

**Figure 2:** Time visualization of the first and second stages of labor of two groups of primiparas (h).

**Figure 3:** Visualization of delivery outcomes of primiparas in two groups (%).

**Figure 4:** Comparison visualization of delivery compliance rate between the two groups (%).

**Table 1:** Comparison of SAS and SDS scores between the two groups of primiparas.

Grouping	SAS	SDS
Reference group	58.71 ± 2.19	59.65 ± 2.15
Observation group	45.12 ± 2.41	43.24 ± 2.08
*t*	7.416	7.358
*P*	0.042	0.041

**Table 2:** Comparison of the first and second stage of labor time of primiparas in the two groups (h).

Grouping	Time of first stage of labor	Time of the second stage of labor
Reference group	9.11 ± 0.25	1.32 ± 0.23
Observation group	8.52 ± 0.29	1.01 ± 0.18

**Table 3:** Comparison of delivery outcomes of primiparas between the two groups (%).

Grouping	Natural childbirth	Parturition lateral incision	Involuntary cesarean section	Voluntary cesarean section
Observation group	30 (69.77%)	5 (11.63%)	4 (9.30%)	4 (9.30%)
Reference group	18 (41.86%)	13 (30.23%)	5 (11.63%)	7 (16.28%)

**Table 4:** Comparison of delivery compliance rate between the two groups (%).

Grouping	*n*	Compliance rate
Observation group	43	95.23%
Reference group	43	78.41%

## Data Availability

The data underlying the results presented in the study are available within the manuscript.
